# Related Factors and a Threshold of the Maximum Neuron-Specific Enolase Value Affecting the Prognosis of Patients with Aneurysmal Subarachnoid Hemorrhage

This article has been retracted.

**DOI:** 10.1155/2022/7596426

**Published:** 2022-05-06

**Authors:** Hao Zhao, Feng Shang, Meng Qi, Yueqiao Xu, Ning Wang, Xin Qu

**Affiliations:** ^1^Department of Neurosurgery, Xuanwu Hospital, Capital Medical University, Beijing 100053, China; ^2^National Center for Neurological Disorders, China; ^3^China International Neuroscience Institute (China-INI), Beijing, China

## Abstract

**Background:**

The prognosis of patients with subarachnoid hemorrhage is influenced by many factors. Neuron-specific enolase (NSE) is a biological marker of neurological damage. This study aimed to determine the related prognostic factors and whether or not the maximum NSE value (NSE_max_) has a threshold between good and poor prognosis in aneurysmal subarachnoid hemorrhage (aSAH).

**Methods:**

A total of 259 patients admitted following aSAH were treated by appropriate methods. Initial neurological severity was evaluated by using the initial Glasgow coma scale and Hunt–Hess grades. NSE plasma concentration was measured during the patient's stay in the neurosurgical intensive care unit, and NSE_max_ was selected for further study. The primary endpoint of the study was Glasgow outcome score (GOS), which was dichotomized as poor outcome (GOS 1–3) or good outcome (GOS 4–5) at discharge.

**Results:**

A poor outcome of patients with aSAH at discharge was associated with mild hypothermia treatment, Hunt–Hess grade, rehemorrhagia, neurogenic pulmonary edema, and pneumonia, which were independent risk factors affecting the prognosis of patients. The best threshold of the maximum value of NSE for poor or good prognosis was 26.255 *μ*g/L (specificity 0.908).

**Conclusions:**

Poor neurological score, pulmonary complications, aneurysm rerupture, and mild hypothermia indicate a poor prognosis. NSE_max_>26.255 *μ*g/L is an independent predicting factor of poor neurological outcome at discharge after aSAH. This threshold value could help clinicians make the appropriate decision and prognosis.

## 1. Introduction

The 30-day mortality rate for aneurysmal subarachnoid hemorrhage (aSAH) is 45%, and almost half of the survivors suffer irreversible brain damage [1]. Relevant complications may occur before and after aSAH treatment, affecting the prognosis of patients. Identifying and quantifying the severity of brain injury to predict prognosis as early as possible are major challenges at present. Initial clinical status determined by Glasgow coma scale (GCS) and Hunt–Hess grade has been associated with prognosis [2, 3]. However, an accurate and direct clinical indicator that can predict the prognosis of patients with aSAH is currently lacking. Recent studies have found that neuron-specific enolase (NSE) is an isoenzyme found in mature neurons, and its expression increases after a stroke or traumatic brain injury, which is related to neurological injury and prognosis [4]. Several trials have reported that NSE is a good predictor of prognosis [5, 6]. During the progression of aSAH, the value of NSE gradually increases and then declines after treatment. However, the maximum value of NSE (NSE_max_) and the relationship with the prognosis of aSAH remain unknown. In this study, we retrospectively analyzed the risk factors of aSAH and hypothesized that the NSEmax threshold has a diagnostic value for the prognosis of aSAH.

## 2. Methods

### 2.1. Study Population and Data Collection

Clinical data of 259 patients with aSAH admitted to the neurosurgical intensive care unit (NICU) of Xuanwu Hospital of the Capital Medical University from March 2016 to March 2019 were randomly selected. This study was approved by the Ethics Committee of Xuanwu Hospital of Capital Medical University (Batch No.: Linyan (2017) No. 024). The inclusion criteria for the patients were as follows: (1) age ≥10 years old; (2) Hunt–Hess grades I–V; (3) spontaneous SAH was confirmed by imaging examination or lumbar puncture; (4) intracranial aneurysm was confirmed by DSA and the aneurysm resulted in SAH; and (5) the family of the patient signed the informed consent and cooperated with the clinical treatment and follow-up. The exclusion criteria were as follows: (1) the patient with aSAH did not undergo NSE examination; (2) previous intracranial aneurysms were treated by clipping or embolization; (3) diagnosis of intracranial aneurysm was unclear; (4) intracerebral hematoma unrelated to the offending aneurysm; (5) the patient was expected to live for less than 1 year due to severe co-occurrence of other systemic diseases; and (6) pregnant or nursing women.

### 2.2. Clinical Features and CT Evaluation

At admission, the patients were assessed by GCS score for clinical neurological severity and then divided into three groups as follows: mild degree of consciousness, GCS = 13–15; moderate degree of consciousness, GCS = 9–12; and severe degree of consciousness, GCS = 3–8. At the same time of admission, the patients were performed brain CT scan and graded by Hunt–Hess grades and then divided into two groups: good grade (I–III) and poor grade (IV–V). At discharge, the neurological outcome was assessed using the Glasgow outcome scale (GOS) score, which was defined as favorable outcome (GOS 4–5) and poor outcome (GOS 1–3).

### 2.3. Clinical Treatment of Aneurysms

Patients included in this study were treated with drug conservative treatment, endovascular embolization surgery, and microsurgical clipping surgery. The patients were transferred to the NICU immediately after the initial admitted and were continuously pumped with nimodipine. Blood pressure was monitored through arteries to ensure that the systolic blood pressure was higher than 130–140 mmHg. Blood sugar and body temperature were monitored daily. With the monitoring of blood gas analysis, carbon dioxide partial pressure (PaCO_2_) was maintained between 35 and 40 mmHg, and SpO_2_ was maintained at more than 97%. Intracranial pressure can be continuously monitored when conditions were permitted. Transcranial ultrasound Doppler examination was performed the next day, and vascular spasm was suspected if intracranial blood flow velocity exceeded 120 cm/s or if the mean transcranial Doppler velocity varied by more than 50 cm/s per day. The dosage of nimodipine was adjusted depending on the condition of vasospasm.

### 2.4. Detection of NSE Level

Arterial samples were collected daily, and NSE was measured immediately after admission to ICU. A small portion of arterial blood was centrifuged in the central laboratory and frozen for further analysis. The sensitivity of NSE in serum was 0.04 *μ*g/L with reference value <18.3 *μ*g/L. In our hospital, no clinical critical care was based on the biomarker level.

### 2.5. Following up

The patients were followed up by using the GOS score. According to the threshold of NSE_max_, patients were systematically divided into two groups (>26.255 and <26.255 *μ*g/L). In each group, we compared the average GOS score at discharge and follow-up period to evaluate the long-term prognosis of the patients.

### 2.6. Statistical Analysis

Statistical analysis of the data was performed using SPSS26.0 (IBM Corp., Armonk, NY, USA). Data are expressed as mean ± standard deviation or count (percentage) as appropriate. Kolmogorov–Smirnov normality test was performed on the continuous data, such as the patient's age, length of stay in ICU, duration of mechanical ventilation (MV), and NSE maximum value. *T* test and nonparametric test were then performed. Variance analysis and *H* test were used for single-factor analysis. One-way ANOVA was performed after homogeneity of variance test for age of patients. Other measurement data were tested by Kruskal–Wallis H nonparametric test. Statistical significance was considered at *P* < 0.05. Categorical variables, such as previous history, gender, Hunt–Hess grading, treatment, pneumonia, GCS score, aneurysm site, endotracheal intubation, mild hypothermia treatment, cerebral infarction, and rehemorrhagia, were reported as proportions and 95% confidential interval (CI) by cross chart chi-square test to detect the effect on the prognosis of patients. Results were performed by odds ratio (OR) with a two-sided *P* < 0.05. The independent risk factors affecting the prognosis of patients were analyzed by binary logistic regression analysis. Statistical significance was considered at *P* < 0.05. Receiver operating characteristic (ROC) curve with the corresponding area under the curve (AUC) and related sensitivity and specificity was used to determine the discriminative ability of NSE_max_ for the prognosis of patients. The Youden index was used for NSE_max_ to calculate the diagnostic threshold value with the best sensitivity and specificity to predict the prognosis of patients. Finally, the patients with aSAH were grouped by the threshold value of NSE_max_, and cross chart chi-square test was adopted to check the validity of the threshold value of NSE_max_.

## 3. Results

### 3.1. Patient General Characteristics

A total of 259 patients with aSAH were enrolled in this study, including 109 males (73.4%) and 150 females (26.6%) (Table 1). A total of 190 patients had a GOS score of 4–5 at discharge, among which 81 were males (75.7%) and 109 were females (71.7%). The average age was 57.59 ± 11.39 years old. A total of 69 patients (10 dead) had a GOS score of 1–3, including 26 males (24.3%) and 43 females (28.3%), with an average age of 60.70 ± 13.23 years old. Statistical results suggested no significant difference in age distribution between the two prognosis groups of aSAH patients at discharge (*P* = 0.065) (Figure 1).

### 3.2. Univariate Logistic Regression Analysis

All patients were admitted to the ICU immediately after surgery, and the longest time staying in the ICU was 139 days, the shortest was 1 day, with an average of 11.16 ± 12.92 days. Patients in the GOS 4–5 group spent an average of 6 days in the ICU, whereas patients in the GOS 1–3 group spent an average of 19.5 days in the ICU (Figure 2). After admission to the ICU, some patients underwent ventilator-assisted breathing after endotracheal intubation, with an average MV duration of 110.16 ± 274.45 h (336.4 ± 446.29 h for patients in the GOS 4–5 group and 26.38 ± 72.96 h for patients in the GOS 1–3 group). The results indicated that the length of ICU stay of patients with aSAH in the GOS 1–3 group was significantly shorter than that in the GOS 4–5 group (*P* < 0.01), and the duration of ventilator ventilation was significantly shorter than that in the GOS 4–5 group. Significant differences were found between the two groups (*P* < 0.01) (Figure 2).

In the group of Hunt–Hess IV–V, 11 (5.8%) patients had a good prognosis, and 26 (37.7%) patients had a poor prognosis. Significant differences were found between the two groups (*χ*^2^ = 42.044, OR = 9.839, 95%CI = 4.512–21.456, *P* < 0.01). In the GCS 3–8 group, 8 (4.2%) patients had a good prognosis, and 27 (39.1%) patients had a poor prognosis. Significant differences were found between the two groups (*χ*^2^ = 54.041, *P* < 0.01). Among the aSAH patients with pneumonia, 52 had a good prognosis (27.4%), and 53 had a poor prognosis (76.8%). Significant differences were found between the two groups (*χ*^2^ = 51.334, OR = 8.791, 95% CI = 4.618–16.733, *P* < 0.01). Among the patients with aSAH undergoing endotracheal intubation, 44 (23.2%) had a good prognosis, and 57 (82.6%) had a poor prognosis. Significant differences were found between the two groups (*χ*^2^ = 75.204, OR = 15.761, 95%CI = 7.765–31.991, *P* < 0.01). Among the patients with aSAH undergoing mild hypothermia treatment, 25 (13.2%) had a good prognosis, and 32 (46.4%) patients had a poor prognosis. Significant differences were found between the two groups (*χ*^2^ = 32.542, OR = 5.708, 95%CI = 3.031–10.751, *P* < 0.01). Among the patients with neurogenic pulmonary edema during treatment, 63 (33.2%) had a good prognosis, and 48 (69.6%) had a poor prognosis. Significant differences were detected between the two groups (*χ*^2^ = 27.397, OR = 4.608, 95%CI = 2.541–8.355, *P* < 0.01). Among the patients with rehemorrhagia, 8 (4.2%) had a good prognosis, and 12 (17.4%) had a poor prognosis. Significant differences were found between the two groups (*χ*^2^ = 12.341, OR = 4.789, 95%CI = 1.866–12.295, *P* < 0.01). All the data are shown in Table 1.

The previous medical history of the patients at admission mainly included diabetes, hypertension, and hyperlipidemia. Statistically speaking, 160 patients had previous medical history, and 99 patients had no previous medical history. The prognosis of patients with or without prior medical history showed no significant difference (*χ*^2^ = 0.033, OR = 0.949, 95%CI = 0.539–1.671, *P* = 0.886). In terms of treatment methods, 25 patients with aSAH received drug conservative treatment, 165 patients received aneurysmal embolization surgeries, and 69 patients received aneurysmal craniotomy clipping surgeries. Different treatments did not have a significant effect on the prognosis of the patients (*χ*^2^ = 2.367, *P* = 0.306). The aneurysms of the enrolled patients were mainly located in the posterior communication artery (110 cases), followed by the anterior communication artery (57 cases). In addition, the aneurysms in 38 cases were located in the middle cerebral artery, and those in 26 cases were located in the vertebral basilar artery. Aneurysms located on other arteries were relatively less. The statistical results showed that aneurysms, whether in the anterior or posterior circulation, were not associated with the prognosis of the patients (*χ*^2^ = 0.811, OR = 1.431, 95%CI = 0.654–3.131, *P* = 0.402). In this study, 42 patients developed delayed cerebral infarction, and no significant difference in prognosis was found between the two prognosis groups (*χ*^2^ = 3.365, OR = 1.904, 95%CI = 0.950–3.817, *P* = 0.085).

### 3.3. Multivariate Binary Logistic Regression and Meta-Analysis Graph

Logistic regression model results suggested that mild hypothermia, Hunt–Hess grade, rehemorhage, neurogenic pulmonary edema, and pneumonia were independent risk factors affecting the prognosis of patients. After adjusting the influencing factors of endotracheal intubation, the probability of poor prognosis in patients with aSAH undergoing mild hypothermia was 3.269 times that of patients not receiving mild hypothermia treatment (*P* <0.01). Patients with severe Hunt–Hess grade of aSAH at admission were 5.674 times more likely to have a poor prognosis than those with mild grade (*P* <0.01). The probability of poor prognosis of aSAH patients with recurrent bleeding during treatment was 4.184 times higher than that of patients without recurrent bleeding (*P* <0.05). aSAH patients with neurogenic pulmonary edema and pneumonia were 2.872 and 3.806 times more likely to have a poor prognosis than those without neurogenic pulmonary edema and pneumonia (*P* <0.01). A meta-analysis graph was established for predicting the prognosis of patients with SAH by integrating independent significant risk factors based on the multivariate binary logistic regression (Figure 3).

### 3.4. NSE_max_ For Outcome in aSAH Patients

Among 259 patients with aSAH, the maximum value of NSE_max_ was 139 *μ*g/L, and the minimum value was 6.56 g/L, with an average value of (11.16 ± 12.924) *μ*g/L (Figure 4). The results indicated that the patients in the poor grade group (GOS 1–3) showed higher NSEmax level than those in the good grade group (GOS 4–5) (*P* < 0.01). ROC curve was used to determine the diagnostic value of NSE to the prognosis of patients.  Figure 5 shows that the AUC of the NSE_max_ value was 0.76, greater than 0.5, and *P* = 0.005 < 0.01, indicating that the NSE_max_ value has a predictive power for the prognosis of patients.

The Youden index of NSE_max_ value was 0.508, and the corresponding NSE_max_ value was 26.255 *μ*g/L, which was taken as the threshold value of the prognosis of patients. If the NSE_max_ value exceeded 26.255 *μ*g/L, the patients were considered to have a poor prognosis, and the corresponding sensitivity and specificity were 0.600 and 0.908. According to the threshold value of NSE_max_, the patients with aSAH were divided into two groups and then statistically analyzed. Results showed that 82.1% of the patients with NSE_max_ values greater than 26.255 *μ*g/L had a poor prognosis (GOS 4–5), whereas only 19.9% of the patients with NSE_max_ values less than 26.255 *μ*g/L had a poor prognosis. Significant differences were found between the two prognosis groups (*P* < 0.01) (Figure 6). This result indicated that the NSE_max_ threshold value of 26.255 *μ*g/L could be used as a diagnostic indicator to predict the prognosis of patients with aSAH.

### 3.5. Follow-Up of Different Group Patients

The GOS score in the group of NSE_max_<26.255 *μ*g/L was significantly higher than that in the group of NSE_max_>26.255 *μ*g/L. In the group of NSE_max_<26.255 *μ*g/L, the GOS scores at follow-up were significantly higher than the GOS scores at discharge (4.381 ± 0.99 vs. 4.451 ± 1.179, *P* = 0.034 < 0.05). However, in the group of NSE_max_>26.255 *μ*g/L, no significant difference was found in GOS scores at discharge and follow-up (2.643 ± 1.162 vs. 2.174 ± 1.497, *P* = 0.12). Instead, some patients had worse GOS scores at follow-up (Figure 7).

## 4. Discussion

The major findings of this respective study are summarized as follows. First, we retrospectively analyzed 259 cases of ICU patients with aSAH and made a comprehensive analysis of various factors affecting the GOS score, which was determined at discharge from the hospital. Second, the value of NSE_max_ was higher in patients with a poor prognosis than in those with good outcomes. Third, the threshold value of NSE_max_ in the blood of patients aSAH patients was calculated to verify its predictive ability on the prognosis of the patients at discharge. To our knowledge, our study is the first to report NSE_max_ threshold for neurological prognosis biomarkers of patients with aSAH.

Endotracheal intubation affects the prognosis of patients. Among patients with poor prognosis, the rate of endotracheal intubation was significantly higher than that without endotracheal intubation (82.6% vs. 23.3%). Among the 10 dead patients, 9 (90%) received endotracheal intubation. Thus, the patient's condition determines whether or not endotracheal intubation should be performed, and patients with endotracheal intubation often have a poor prognosis. Large multicenter population studies have shown that 10%–15% of inpatients require endotracheal intubation and MV. Among them, SAH accounted for 29% of the cases [7]. Stroke patients undergoing MV had a poor prognosis, with hospitalization mortality ranging from 53% to 57% [8] and one-year mortality ranging from 60% to 92% [9–13]. Endotracheal intubation and MV appeared to be major predictors of mortality. Among 31,300 patients from the USA with ischemic stroke, the risk ratio (HR) for 30-day mortality was 5.6 [14]. In another population-based study of 798,255 stroke patients, the likelihood of discharge decreased from 37% to 12% due to endotracheal intubation and MV. Although endotracheal intubation and MV are considered indicators of clinical severity, the causes of endotracheal intubation may be associated with potentially rapidly progressing conditions (such as epileptic persistence, pneumonia, septicemia, or hydrocephalus) that affect the patient's prognosis [15].

Previous medical history did not influence the prognosis of patients. In this study, the distribution of past history of patients in different groups was basically balanced, indicating that the patients had a past history at the time of onset or not, which could not predict the prognosis of patients. However, the existence of past history often complicates the treatment process. In future studies, we will subdivide the past history of patients and further investigate the correlation with the prognosis of patients. The higher the Hunt–Hess grade at admission, the worse the prognosis. In general, Hunt–Hess grades for IV–V patients indicate mild hypothermia therapy, and the patients' prognosis is poor. In addition, the probability of related complications increases in patients undergoing mild hypothermia treatment, which also affects the prognosis of patients.

The present study found that pulmonary infection could lead to poor prognosis. Prolonged bed stay could lead to lung infections, and the utilization of ventilators could aggravate pneumonia. Therefore, improving the pulmonary condition of aSAH patients is highly important. Neurogenic pulmonary edema is a clinical syndrome characterized by acute pulmonary edema after central nervous system injury. It has two possible mechanisms of pathogenesis. One is the blood circulation dynamics theory, and the other is the pulmonary vascular permeability theory. The development of neurogenic pulmonary edema is associated with deteriorating clinical outcomes. In one study, the fatality rate for neurogenic pulmonary edema was up to 59%, and only 23% of patients had a good prognosis [16–18]. In our hospital, routine pulmonary ultrasonography was taken to detect the occurrence of pulmonary edema as soon as possible and monitor the changes in pulmonary edema. For patients with severe ARDS, prone ventilation can improve the patient's breathing and often achieve satisfactory results.

In the present study, rehemorrhage was one of the strongest predictors of poor outcome, which was similar to previous studies [19]. Earlier studies had shown that within 24 h of the initial aneurysmal SAH, about 4% of patients would rebleed, with a 1%–2% chance of rebleeding every day for the next 14 days. If hyperacute rebleeding occurring within less than 8 h was included, the incidence of rebleeding within the first 24 h was probably closer to 12%. Early angiography (<3 hours) and early treatment of aneurysms by microsurgical clipping or coil embolization are critical to reduce the incidence of rebleeding. A short-term antifibrinolytic therapy reduces rebleeding and possibly improves outcomes, but current data suggest that this conclusion is inconclusive.

NSE is an enolization enzyme isozyme specifically distributed in neurons and a few neuroendocrine cells under normal circumstances. NSE has small quantity in blood and cerebrospinal fluid, but it can be released into the cerebrospinal fluid by incomplete cell membrane and then into the blood through the ruptured blood–brain barrier when brain injury, ischemia, and edema occur. NSE can be used as a reliable indicator for the diagnosis of neurocyte damage with high specificity and can further reflect the degree of brain damage. After SAH occurs, NSE will be released from the damaged neurocyte into the cerebrospinal fluid, peak within 24 h after bleeding, and then decline progressively. NSE will peak at the second time 3–4 days after SAH, which is related to secondary brain injury. NSE can hardly cross the blood–brain barrier. Thus, the peak time of NSE in serum is usually 2–3 days later than that in cerebrospinal fluid. Serum NSE levels rise because the blood–brain barrier is broken before they enter the blood. Thus, a high or low NSE is often a proxy for the severity of brain damage.

We collected all NSE values of the patients during hospitalization and selected NSE_max_ for statistical analysis, confirming the important predictive value of this biomarker. The NSE_max_ value was high in the poor prognosis group. Previous studies proposed the mean value of NSE during NICU stay to assess the prognosis of patients with aSAH. However, it is difficult to handle in clinical practice. NSE value is a continuously changing number. Herve Quintard et al. evaluated biomarkers within 7 days following SAH to obtain an early parameter to guide the clinician to determine prognosis. Evaluating NSE for a long period might produce different results [20]. Therefore, the definition of a cutoff value of NSE during aSAH could be helpful for clinicians to make a decision. Our results suggest that NSE_max_ is an important tool to help clinicians supply a suggestion on the patient's prognosis and to make decisions about prolonging or withdrawing aggressive treatment. In our study, the NSE_max_ value was related to the GOS score of patients at discharge. The NSE_max_ value greater than 26.255 *μ*g/L was the critical value for the poor prognosis of patients. Many relevant studies also provided evidence in this regard. Moritz found that within 24 h after SAH, the NSE level in cerebrospinal fluid and serum temporarily increases and then gradually decreases. If the NSE level no longer increases, the prognosis of patients would be good. We followed up the neurological recovery after discharge. A previous study found that some patients experience delayed recovery after discharge [21]. In the present study, neurological recovery obviously improved in the group of NSE_max_<26.*μ*/L but surprisingly declined in the group of NSE_max_>26.255 *μ*g/L. Therefore, the threshold of NSE_max_ was a good prognostic indicator in patients with aSAH. This finding has a great significance to guiding our clinical work.

This study has several limitations. First, it is a retrospective analysis of cases. Some data for NSE values were missing, so large prospective studies are needed in the future to confirm the usefulness of continuous NSE measurements and evidence-based conclusions in predicting the neurological outcomes in patients with SAH. Second, the diagnosis of delayed cerebral infarction was retrospectively analyzed. Vasospasm is the primary reason for delayed cerebral infarction, but the diagnostic capacity of transcranial Doppler as a noninvasive monitoring tool for cerebral vasospasm is limited [22, 23]. In addition, cerebral MRI is not routinely used to detect silent infarction after SAH, which may have limited the detection of delayed cerebral infarction in this study. Third, NSE levels may be elevated in patients with chronic inflammatory and neurodegenerative diseases. In this study, we could not exclude patients with mild or undiagnosed diseases.

## 5. Conclusions

Prevention of aSAH risk factors contributes to a good prognosis when patients are discharged from the hospital. The need to determine accurate biomarkers for prognosis assessment is essential to improve care in the critically ill patients. Factually, NSE_max_ may be a reliable predicted value of prognosis in aSAH. Definition of the threshold value of NSE_max_ (26.255 *μ*g/L) could help physicians estimate the prognosis according to the predictive values of biomarkers, either at patients' discharge or during follow up.

## Figures and Tables

**Figure 1:** Age distribution of patients in different aSAH prognosis groups.

**Figure 2:** ICU stay and mechanical ventilation duration of aSAH patients in the GOS 1–3 and GOS 4–5 groups.

**Figure 3:** Meta-analysis graph based on the binary logistic regression model.

**Figure 4:** Maximum value of NSE was significantly different between two prognosis groups.

**Figure 5:** ROC curve, area under curve (AUC), and diagnostic threshold (Yoden index) of NSE_max_ in aSAH patients.

**Figure 6:** Distribution of different prognosis of aSAH patients with the highest NSE value greater than 26.255 *μ*g/L and NSE less than 26.255 *μ*g/L.

**Figure 7:** Change of GOS scores in two different groups at discharge and during follow up.

**Table 1:** Baseline characteristics among two GOS groups.

Variables	GOS scores at discharge		*χ* ^2^	OR	95% CI	*P*
	GOS 4-5	GOS 1-3				
Sex (*n*, %)						
Male	81 (42.6%)	26 (37.7%)	0.512	0.814	0.462-1.432	0.568
Female	109 (57.4%)	43 (62.3%)				
Hunt–Hess grade (*n*, %)						
Good	179 (94.2%)	43 (62.3%)	42.044	9.839	4.512-21.456	<0.01
Poor	11 (5.8%)	26 (37.7%)				
Intervention (n, %)						
Medical	18 (9.5%)	17 (10.1%)	2.367			0.306
Endovascular	126 (66.3%)	39 (56.5%)				
Microsurgical clipping	46 (24.2%)	23 (33.3%)				
GS score (*n*, %)						
Mild (12-15)	162 (85.3%)	34 (49.3%)	54.041			<0.01
Medium (9-1)	20 (10.5%)	8 (11.6%)				
Severe (3–8)	8 (4.2%)	27 (39.1%)				
Location of aneurysm (n, %)						
Anterior circulation	166 (88.3%)	58 (84.1%)	0.811	1.431	0.654-3.131	0.402
Posterior circulation	22 (11.7%)	11 (15.9%)				
Past medical history (*n*, %)						
w/o	72 (37.9%)	27 (39.1%)	0.033	0.949	0.539-1.671	0.886
W	118 (62.1%)	42 (60.9%)				
Pneumonia (*n*, %)						
w/o	138 (72.6%)	16 (23.2%)	51.334	8.791	4.518-16.733	<0.01
W	52 (27.4%)	53 (76.8%)				
Endotracheal intubation (*n*, %)						
w/o	146 (76.8%)	12 (17.4%)	75.204	15.761	7.765-31.991	<0.01
W	44 (23.2%)	57 (82.6%)				
Mild hypothermia (*n*, %)						
w/o	165 (86%)	37 (53.6%)	32.542	5.708	3.031-10.751	<0.01
W	25 (13.2%)	32 (46.4%)				
Neurogenic pulmonary edema (*n*, %)						
w/o	127 (66.8%)	21 (30.4%)	27.397	4.608	2.541-8.355	<0.01
W	63 (33.2%)	48 (69.6%)				
Cerebral infarction (*n*, %)						
w/o	164 (86.3%)	53 (76.8%)	3.365	1.904	0.950-3.817	0.085
W	26 (13.7%)	16 (23.2%)				
Rehemorrhagia (*n*, %)						
w/o	182 (95.8%)	57 (82.6%)	12.341	4.789	1.866-12.295	<0.01
W	8 (4.2%)	12 (17.4%)				

## Data Availability

The data used to support the findings of this study are available from the corresponding author upon request.

## Abbreviations

AUC: Area under the curve
CI: Confidential interval
GCS: Glasgow coma scale
GOS: Glasgow outcome score
MV: Mechanical ventilation
NICU: Neurosurgical intensive care unit
NSE: Neuron-specific enolase
OR: Odds ratio
ROC: Receiver operating characteristic.
